The article "miR-92b-3p Exerts Neuroprotective Effects on Ischemia/Reperfusion-Induced Cerebral Injury via Targeting NOX4 in a Rat Model" was retracted in 2023. Reasons: signs of a paper mill; compromised peer review; unreliable results or conclusions.

# miR-92b-3p Exerts Neuroprotective Effects on Ischemia/Reperfusion-Induced Cerebral Injury via Targeting NOX4 in a Rat Model

**DOI:** 10.1155/2022/3494262

**Published:** 2022-03-30

**Authors:** Yongpan Huang, Jiayu Tang, Xiaojuan Li, Xian Long, Yansong Huang, Xi Zhang

**Affiliations:** ^1^School of Medicine, Changsha Social Work College, Changsha, Hunan, China; ^2^Department of Neurology, Brain Hospital of Hunan Province, Changsha, Hunan, China; ^3^Hunan Brain Hospital, Clinical Medical School of Hunan University of Chinese Medicine, Changsha, Hunan, China

## Abstract

The necessity to increase the efficiency of organ preservation has pushed researchers to consider the mechanisms to minimize cerebral ischemia/reperfusion (I/R) injury. Hence, we evaluated the role of the miR-92b-3p/NOX4 pathway in cerebral I/R injury. A cerebral I/R injury model was established by blocking the left middle cerebral artery for 2 h and reperfusion for 24 h, and a hypoxia/reoxygenation (H/R) model was established. Thereafter, cerebral I/R increased obvious neurobiological function and brain injury (such as cerebral infarction, apoptosis, and cell morphology changes). In addition, we noted a significant decrease in the expression of miR-92b-3p, as well as increases in apoptosis and oxidative stress and an increase in NOX4. Furthermore, overexpression of miR-92b-3p blocked the inhibitory effect of miR-92b-3p on the expression of NOX4 and the accumulation of oxygen-free radicals. Bioinformatics analysis found that NOX4 may be the target gene regulated by miR-92b-3p. In conclusion, the involvement of the miR-92b-3p/NOX4 pathway ameliorated cerebral I/R injury through the prevention of apoptosis and oxidative stress. The miR-92b-3p/NOX4 pathway could be considered a potential therapeutic target to alleviate cerebral I/R injury.

## 1. Introduction

Stroke is a type of cerebrovascular disease associated with high rates of disability and an increasing incidence and is divided into ischemic and hemorrhagic stroke. Ischemic stroke, also known as cerebral infarction, accounts for approximately 80% of all strokes [1–3] and is a disease of acute/onset focal/hemispheric brain dysfunction caused by ischemic factors that last for more than 24 hours. Ischemic stroke is mainly due to insufficient blood supply to the brain caused by cerebral artery occlusion, resulting in local cerebral tissue ischemia and hypoxia. Neuronal cells in the brain tissue exhibit energy or ion pump obstacles [4–6] and rapidly develop reversible or irreversible neuronal damage; therefore, subsequent reperfusion of acute ischemic stroke is essential for neuronal cell rescue [7]. However, experimental and clinical evidence has shown that restoration of perfusion, the contradiction of increased damage in the short term, often leads to reperfusion injury [8–14]. Such an injury is related to impaired blood flow, cellular necrosis, and vascular dysfunction, and the mechanism is associated with calcium overload, intense inflammatory response, and oxidative stress. Excessive production of active oxygen and/or decreased antioxidant capacity leads to deleterious consequences. Clinical and experimental studies have provided substantial evidence that reactive oxygen species (ROS) can be produced during cerebral ischemia/reperfusion (I/R), of which the amount produced at the beginning of reperfusion is the most significant [15, 16]. ROS can assault neuronal cells by directly attacking the cell membrane and various macromolecular substances (such as nucleic acids and proteins), causing neuronal cell necrosis or activating redox signaling pathways to induce neuronal cell apoptosis [16, 17]. Increased reactive oxygen production during cerebral I/R is associated with upregulation of certain prooxidase gene expression and increased activity. A large number of studies have shown that NOX-derived active oxygen plays an important role in oxidative stress injury in cerebral I/R [18]. Recent studies have found that both NOX2 and NOX4 are upregulated in I/R rat brain tissues, while NOX1 has no significant changes, suggesting that NOX2 and NOX4 are mainly involved in oxidative stress injury during cerebral I/R [19].

miRNAs are a type of endogenous noncoding small RNA with a length of 20–24 nucleotides that are complementary to the 3′ untranslated regions (3′UTRs) of the target gene mRNA and function by degrading the target gene mRNA or inhibiting its translation, decreasing the expression levels of target genes [20, 21]. Once the expression levels of miRNAs decrease, their inhibitory effects on the expression of target genes decrease, and the expression levels of target genes increase. Recent studies have demonstrated that the expression levels of various miRNAs are significantly altered, which may be involved in the pathophysiological process of I/R injury, including miR-497, miR-1, and miR-181, which are related to neuroprotection [22, 23]. Recently, a study has shown that miR-92b-3p, may be involved in the occurrence of oxidative stress injury during cerebral I/R induced by NOX4 overexpression, which eventually leads to the accumulation of oxygen free radicals and the death of neuronal cells from oxidative stress injury [24]. This study showed that miR-92b-3p was significantly decreased in a cerebral I/R injury rat model.

The article "miR-92b-3p Exerts Neuroprotective Effects on Ischemia/Reperfusion-Induced Cerebral Injury via Targeting NOX4 in a Rat Model" was retracted in 2023. Reasons: signs of a paper mill; compromised peer review; unreliable results or conclusions.

Using the bioinformatics software TargetScan and miRBase, NOX4 gene brain-specific or brain-rich targeted miRNAs were predicted, and it was initially determined that miR-92b-3p may be a miRNA that specifically regulates NOX4. The present study is aimed at investigating the role and possible mechanism of the miR-92b-3p/NOX4 pathway in oxidative damage in the cerebral I/R rat model and a H/R neuronal cell injury model.

In addition, we showed that nicotinamide adenine dinucleotide phosphate (NADPH) oxidase 4 (NOX4) was a target of miR-92b-3p, and NOX4 inhibition by GLX351322 protected against oxidative stress in cerebral I/R rat model and a H/R neuronal cell injury model, which indicated that miR-92b-3p/NOX4 were potential therapeutic targets for ischemic stroke.

## 2. Materials and Methods

### 2.1. Animal Experiments

Male Sprague–Dawley rats weighing 250–300 g were purchased from Beijing Vital River Laboratory Animal Technology Co., Ltd. (2020–00B1) and were kept in the Animal Experiment Center of Central South University. The rats were given ad libitum access to food and water. All experiments were carried out according to the guidelines for the Care and Use of Laboratory Animals (NIH Publication No. 85–23, revised 1996) and were approved by the Brain Hospital of Hunan Province Animal Care and Use Committee. The animals were randomly divided into the control (*n* = 10), sham (*n* = 10), and cerebral I/R (*n* = 40) groups. All the animals were kept in a temperature and humidity-controlled environment with a 12 h light/dark cycle at 22-25°C, with 50-65% humidity and free access to food and water.

### 2.2. Cell Culture

Neural cells (SH-SY5Y) were provided by the Shanghai Experimental Cell Center, Chinese Academy of Sciences. We followed the methods of Huang et al. [25]. SH-SY5Y cells were authenticated by short tandem repeat identification. SH-SY5Y cells were cultured in DMEM supplemented with 10% FBS, 100 m/ml penicillin, and 100 m/ml streptomycin and were maintained in a humidified atmosphere of 5% CO_2_ at 37°C. The medium was changed every 2 days. All assays consisting of appropriate controls were performed in triplicate and repeated on three separately initiated cultures.

### 2.3. Experimental Protocol

#### 2.3.1. Preparation and Experimental Grouping of the Rat Cerebral I/R Model

The tether thread used to construct the cerebral I/R model was purchased from Beijing Shandong Biotechnology Co., Ltd. The head diameter of the tether thread was 0.40 ± 0.02 mm, and it was marked black at a distance of 2.0 cm from the head. We followed the methods of Zhang et al. [26]. After all the animals were anesthetized by an intraperitoneal injection of pentobarbital sodium (30 mg/kg), the neck hair was cut, 75% medical-grade alcohol was used to disinfect the skin, the skin of the neck was cut with ophthalmic scissors, the muscle was carefully peeled away, and the left common carotid artery (CCA) was exposed and separated from the external carotid artery (ECA) and the internal carotid artery (ICA). The proximal ends of the CCA and ECA were ligated with the prepared thread, a spare silk thread was placed at the distal end of the CCA to tighten the nylon thread and blood vessel blocking blood flow, and the ICA was temporarily clamped with an arterial clip. Ophthalmic scissors were utilized to cut a small opening in the blood vessel wall between the proximal and distal wires of the CCA. After the blood flow in the blood vessel was clear, the MCAO plug wire was inserted into the internal carotid artery along with the vascular opening, the wire was tightened, and the ICA was released. Ophthalmic forceps were utilized to send the tether line along the ICA intracranially until the marked position on the tether line reached the appropriate location under the bifurcation of the external carotid artery (ECA) and the internal carotid artery (ICA). Counting from the bifurcation, the insertion depth was approximately 18–20 mm. After blocking the blood flow for 2 h, the plug was pulled out to achieve reperfusion. At the same time, the spare thread was ligated to the CCA telecentric end, and the skin was sewn. After reperfusion for 24 h, the animals were well treated.

The article "miR-92b-3p Exerts Neuroprotective Effects on Ischemia/Reperfusion-Induced Cerebral Injury via Targeting NOX4 in a Rat Model" was retracted in 2023. Reasons: signs of a paper mill; compromised peer review; unreliable results or conclusions.

#### 2.3.2. Evaluation of Neurological Scoring

Neurological function was determined by a blinded investigator at 24 h after cerebral ischemia according to a previously described protocol for neurological scoring [26, 27]. The scoring was evaluated by the following standards: 0 points, the rats behaved normally; 1 point, the rats could not fully stretch their left forefeet; 2 points, the rats spun in space; 3 points, the rats fell to the left direction; and 4 points, the rats could not move autonomously and fully lost consciousness.

#### 2.3.3. 2,3,5-Triphenyltetrazolium Chloride Staining (TTC Staining)

We followed the methods of Zhang et al. [26]. The tissue sections were put in 1% triphenyl-2,3,5-tetrazolium chloride (TTC) (cat. T8877: Sigma-Aldrich; Merck KGaA) at 37°C for 30 min. The tissue sections were moved every 5 min, followed by washing with ddH_2_O 3 times. Then, photographs were collected for further analysis. The size of the infarct area (white) was evaluated using the ImageJ software.

#### 2.3.4. Hematoxylin and Eosin (HE) Staining

Brain tissues were collected and fixed in 4% paraformaldehyde (cat. 158127: Sigma-Aldrich; Merck KGaA) and dehydrated until transparent. The tissues were embedded in paraffin and then cut into thin slices (4 *μ*m) for HE staining. Morphological changes in brain tissues were observed under an optical microscope (×200) in 3 random areas.

The article "miR-92b-3p Exerts Neuroprotective Effects on Ischemia/Reperfusion-Induced Cerebral Injury via Targeting NOX4 in a Rat Model" was retracted in 2023. Reasons: signs of a paper mill; compromised peer review; unreliable results or conclusions.

#### 2.3.5. TUNEL Assay

TUNEL staining was performed as previously described [26, 28]. Briefly, brain slices were fixed in 4% paraformaldehyde solution for 0.5 hours at room temperature. Then, the slices were incubated with a methanol solution containing 0.2% H_2_O_2_ for another 0.5 hours to block the activity of endogenous peroxidase. Then, the TUNEL reaction mixture was added and incubated at 37°C for 60 minutes. Finally, 3 fields were randomly selected to take photographs by microscopy. The final results were quantified as (TUNEL − positive cells)/(total cells) × 100%.

#### 2.3.6. Preparation and Experimental Grouping of a Hypoxia-Reoxygenation (HR) Model of a Neural Cell Line (SH-SY5Y) and Transfection

SH-SY5Y cells were inoculated into the culture plate, cultured with a normal medium containing 10% fetal bovine serum under the conditions of 95% air, 5% CO_2_, and 37°C to 70%-80% fusion growth, and then the medium was replaced with medium containing 1% fetal bovine serum to synchronize for 12 h. After the synchronization was completed, the medium was replaced with a hypoxic medium (balanced salt solution) under 95% N_2_ and 5% CO_2_ for 4 h (hypotrophic medium only needs to cover the minimum volume of the layer cells to prevent the cells from becoming dehydrated), and the medium was replaced with normal medium without serum in 95% air, 5% CO_2_, and 37°C for reoxygenation for 24 h. Then, SH-SY5Y cells were inoculated into a 24-well plate and transfected with 100 nM miR-92b-3p inhibitor (miR-92b-3p group) or the negative control (miR-NC group) using Lipofectamine 2000 (Invitrogen, Carlsbad, CA, USA) according to the manufacturer's instructions. After 48 h, the cells were collected for subsequent analysis.

#### 2.3.7. Apoptosis Assay

SH-SY5Y cells were cultured in a 6-well plate, washed with phosphate-buffered saline (PBS) (cat. ST476: Sigma-Aldrich; Merck KGaA), and fixed with 70% ethanol. Then, PBS (pH 7.4) containing Annexin V/PI, RNase, EDTA, and Triton X-100 was added to the cells, and the cells were incubated at 37°C for 30 min, followed by incubation at 4°C for 1 h in the dark. The apoptosis rate was detected using a flow cytometer (Becton, Dickinson, Franklin Lakes, NJ, USA).

#### 2.3.8. Western Blotting

At 24 h after reperfusion, the brain tissues were harvested. Total protein was extracted with RIPA lysis buffer from ischemic brain tissues, transferred onto a PVDF membrane (Millipore, Billerica, MA, USA), sealed with 5% skim milk powder, and incubated with the anti-NOX4 primary antibody (cat. ab3517: Abcam, Cambridge, UK) overnight. Then, the protein was incubated again with the HRP-coupled secondary antibody, followed by analysis using an ECL system (Fusion FX7).

The article "miR-92b-3p Exerts Neuroprotective Effects on Ischemia/Reperfusion-Induced Cerebral Injury via Targeting NOX4 in a Rat Model" was retracted in 2023. Reasons: signs of a paper mill; compromised peer review; unreliable results or conclusions.

#### 2.3.9. Detection of Changes in miRNA and mRNA Levels Using Quantitative Reverse Transcription-Polymerase Chain Reaction (qRT-PCR)

Total RNA was extracted from cells using TRIzol reagent and quantified using a NanoDrop ND-2000 (Thermo, Waltham, MA, USA). The RNA was reverse transcribed using reverse transcriptase. Then, the miR-92b-3p/U6 and NOX4/GAPDH levels were quantified using the CFX96 real-time PCR detection system (Bio-Rad, Hercules, CA, USA). The primer sequences in qRT-PCR are shown in Table 1.

#### 2.3.10. Prediction and Analysis of Target Genes

The target genes of miR-92b-3p were predicted using TargetScan, and they were uploaded to Metascape for enrichment analysis. TargetScan21 is an online database specialized in analyzing mammalian miRNA target genes, and it has multiple sublibraries (TargetScan Human, TargetScan Mouse, TargetScan Fly, TargetScan Worm, and TargetScan Fish) according to different species. Metascape22 integrates many authoritative data resources (GO, KEGG, UniProt, and DrugBank) so that it is capable of not only pathway enrichment and biological process annotation but also gene-related protein network analysis and related drug analysis.

#### 2.3.11. Luciferase Activity Assay

The relative luciferase activity was examined by using the Promega Bright-N-Glo system (Promega, USA). The miR-92b-3p overexpression construct and control vector was obtained from Shanghai Genchem (China). The 3′UTR of NOX4 was amplified using the following primers: forward 5′-CCG CTC GAG AAC CTT AGG AGA CTA CTG GGG ACT TT-3′, reverse 5′-TCC GAA GAT CTC CAT CAA AAT TCG TGA TTT AAG ATT T-3′. The polymerase chain reaction (PCR) product was cloned into the pGL3-CMV-LUC-MCS vector (Shanghai Genomeditech, China) and verified by sequencing to create the recombinant plasmid pGL3-NOX4-3′UTR. The mutation was created by PCR using the following primers: fragment 1 forward 5′-CCG CTC GAG AAC CTT AGG AGA CTA CTG GGG ACT TT-3', reverse 5′-CAG TTT CAA CCT GGG AGT GTT TGC CTG GAG CCT AT-3′; fragment 2 forward 5′-AGG CAA ACA CTC CCA GGT TGA AAC TGT AGC ACA AA-3′, reverse 5′-TCC GAA GAT CTC CAT CAA AAT TCG TGA TTT AAG ATT T-3′. The PCR products were mixed as the template and amplified with PCR to generated the mutant 3′UTR of Nox4 (pGL3-NOX4-3′UTR mutant), which was verified by sequencing. SH-SY5Y cells were transfected with miR-92b-3p of control vector and wild-type or mutant NOX4 3′UTR plasmid with phRL-CMV Renilla for 48 h, and relative luciferase activity was examined. Sequences of primers for quantitative RT-PCR using miR-92b-3p primers are as follows: forward 5′-GTC CGC TAT TGC ACT CGT CCC GGC CTC C-3′, reverse 5′-GTG CGT GTC GTG GAG TC-3′; U6 forward 5′-GTC CGC GTG CTC GCT TCG GCA GC-3′, reverse 5′-GTG CGT GTC GTG GAG TC-3′; and GAPDH forward 5′-AGG TCG GTG TGA ACG GAT TTG-3′, reverse 5′-TGT AGA CCA TGT AGT TGA GGT CA-3′.

The article "miR-92b-3p Exerts Neuroprotective Effects on Ischemia/Reperfusion-Induced Cerebral Injury via Targeting NOX4 in a Rat Model" was retracted in 2023. Reasons: signs of a paper mill; compromised peer review; unreliable results or conclusions.

#### 2.3.12. Hoechst 33258 Staining

For the detection of apoptosis, Hoechst 33258 staining was performed as previously described [29]. After H/R, the culture solution was exhausted and then fixed for 10 min. The cultures were then washed twice with PBS, 3 min each time. After aspirating the liquid, 0.5 ml of Hoechst 33258 staining solution (cat. C1018: Beyotime Biotechnology, China) was added to stain the cells for 5 min in the dark. After 5 min, the staining solution was removed, and the cells were washed twice with PBS in the dark for 3 min each time. After aspirating the liquid, 0.8 ml of PBS was added for blocking, and one drop of antifluorescence quencher was added to each well. The blue cell nuclei were the targeted positive cells. The apoptosis rate was detected using a fluorescence microscope (the excitation wavelength was 350 nm, and the emission wavelength was 460 nm). The results are expressed as a percentage of the number of positive cells to the total number of cells.

#### 2.3.13. Methyl Thiazolyl Tetrazolium (MTT) Assay

At 24 h after transfection, the cells were inoculated into a 96-well plate (3 × 103 cells/well), with five replicates in each group. MTT buffer (cat. 11465007001: Roche, Switzerland) was added to the 96-well plate, and the cell viability was detected at 0, 24, 48, and 72 h. The optical density at 570 nm (OD570) was measured using a microplate reader (Bio-Rad, Hercules, CA, USA).

#### 2.3.14. Determination of Flow Cytometry

SH-SY5Y cells were cultured in a 6-well plate, washed with phosphate-buffered saline (PBS), and fixed with 70% ethanol. Then, PBS (pH 7.4) containing Annexin V/PI, RNase, EDTA, and Triton X-100 was added to the cells, and the cells were incubated at 37°C for 30 min, followed by incubation at 4°C for 1 h in the dark. The apoptosis rate was detected using a flow cytometer (Becton, Dickinson, Franklin Lakes, NJ, USA).

#### 2.3.15. Statistical Analysis

All data were statistically analyzed using the SPSS 21.0 software. Data are expressed as the mean ± standard error. ANOVA and Bonferroni's multiple comparison *t-*test analysis was used to compare the means of multiple groups. *P* < 0.05 was considered statistically significant.

## 3. Results

### 3.1. Cerebral I/R Caused Cerebral Infarction and Neurobiological Damage in Rats

The neurobiological scores showed that the control group and the sham operation group had essentially no neurological deficits (score of 0). Compared with the control group, there was obvious neurobiology indicating functional injury in the cerebral I/R group (*P* < 0.01); the degree of injury was mostly above moderate (score > 2), and a small number of rats died during model preparation due to severe assaults (Figure 1(a)).

The article "miR-92b-3p Exerts Neuroprotective Effects on Ischemia/Reperfusion-Induced Cerebral Injury via Targeting NOX4 in a Rat Model" was retracted in 2023. Reasons: signs of a paper mill; compromised peer review; unreliable results or conclusions.

TTC staining showed that the sections from the control and sham groups were stained red, indicating that there was no damage to the brain tissue and no infarcts occurred; conversely, the ischemic hemisphere of the cerebral I/R group showed an obvious white stained area (infarction area), indicating that the brain tissue was severely damaged and that related metabolic enzymes were lost or inactivated (Figure 1(b)). Infarct volume statistics showed that the cerebral infarction volume in the I/R group reached 0.4 cm^3^, which was significantly different from those in the control and sham groups (0 infarctions) (Figure 1(c)) (*P* < 0.01). The infarct area coincided with the blood supply range of the middle cerebral artery, indicating the success of the I/R model.

HE staining showed that the control and sham groups had clear and complete organizational structures, dense cell distribution, normal round or oval nuclei, and normal cell morphology, indicating that there was no release of tissue hydrolase. The results of cerebral I/R injury included a loosened arrangement, degenerated neurons and necrosis, a contracted nucleus, a no longer visible nucleolus, and a large cavity in the intercellular space (Figure 1(d)).

### 3.2. Cerebral Ischemia/Reperfusion Induces Apoptosis in Rat Brain Tissue

We evaluated the apoptosis of tissue cells after cerebral I/R by TUNEL immunohistochemistry and detected caspase-3 enzyme activity. The results of the TUNEL staining showed that after cerebral I/R, the neuronal cells of brain tissues showed obvious DNA breaks, indicated from the staining with dark blue to blue-violet particles in the cell nuclei, that is, TUNEL-positive cells. Few TUNEL-positive cells in the brain tissues of the control and sham groups were observed (Figure 2(a)). The statistics of TUNEL-positive cells showed that the number of TUNEL-positive neurons in the cerebral I/R group was as high as 600/mm^2^ compared with the control and sham groups (*P* < 0.01) (Figure 2(b)).

Compared with the control and sham groups, cerebral I/R significantly increased caspase-3 activity in brain tissue (*P* < 0.05), and these results were consistent with the TUNEL staining results (Figure 2(c)).

### 3.3. Expression Changes of miRNAs Rich in Brain Tissue after I/R

Eight brain tissue-specific miRNAs and 3 brain tissue-rich miRNAs were selected for RT-PCR analysis to measure their expression levels in brain tissue and plasma after I/R. The results showed that the expression levels of miR-126a, miR-29b, miR-188, miR-92b-3p, miR-150b, and miR-532 were significantly downregulated after I/R (Figure 3), while only the expression level of miR-92b-3p was significantly downregulated in rat plasma, suggesting that miR-92b-3p may have important significance in cerebral I/R injury.

The article "miR-92b-3p Exerts Neuroprotective Effects on Ischemia/Reperfusion-Induced Cerebral Injury via Targeting NOX4 in a Rat Model" was retracted in 2023. Reasons: signs of a paper mill; compromised peer review; unreliable results or conclusions.

### 3.4. NOX4 Served as a Direct Target of miR-92b-3p

We intended to verify the functional targets of miR-92b-3p to further confirm the association between miR-92b-3p and NOX4. We focused on miR-92b-3p downregulation in brain tissues and plasma levels after I/R using bioinformatics methods to predict the target genes directly affected by miR-92b-3p. TargetScan software analysis found that among the target genes affected by miR-92b-3p, NOX4 is closely related to cerebral I/R injury (Figure 4(a)). Additionally, miRBase software analysis found that miR-92b-3p was also included in the target miRNAs of NOX4 (TECPR2) (Figure 4(b)). A bidirectional bioinformatics analysis indicated that NOX4 may be the target gene of miR-92b-3p. The sequence, score, and probability of its interaction are shown in Figure 4(c). To confirm the prediction, a dual-luciferase reporter assay was operated on 293T cells cotransfected with a reporter vector of 3′UTR fragments of NOX4 containing either the wild-type or the mutated putative miR-92b-5p binding site and miR-92b-3p mimics. The findings indicate that overexpression of miR-92b-3p decreased the luciferase activity of the reporter vector containing the wild-type NOX4 3′UTR and not mutated NOX4 3′UTR in miR-92b-3p overexpression cells. These results implied that miR-92b-3p bound to 3′UTR of NOX4 at the predicted binding site. Next, the impact of miR-92b-3p on NOX4 expression was measured. We found that overexpression of miR-92b-3p downregulated the NOX4 expression in mRNA and protein levels. These results suggested that NOX4 was a direct target gene of miR-92b-3p.

### 3.5. Changes in miR-92b-3p and NOX4 Expression after I/R

RT-PCR was used to determine the expression levels of miR-92b-3p and NOX4 mRNA. As shown in Figures 5(a) and 5(b), the results showed that, compared with the control and sham groups, I/R downregulated miR-92b-3p expression in tissues and the plasma, while NOX4 mRNA expression was noticeably upregulated (Figure 5(c)). Western blotting results showed that after I/R, NOX4 protein expression in brain tissue was significantly upregulated (Figure 5(d)).

### 3.6. Exogenous miR-92b-3p Mimic Inhibited NOX4 Expression and ROS Levels

To confirm the role of miR-92b in the regulation of NOX4 expression, a H/R injury model of a nerve cell line (SH-SY5Y) was established to simulate the situation in vivo, and cells were treated with miR-92b mimics. As shown in Figure 6(a), transfection with the miR-92b-3p mimics significantly upregulated the expression level of miR-92b-3p in SH-SY5Y cells, indicating the successful design and synthesis of the miR-92b mimics. After H/R, the expression of miR-92b-3p was significantly downregulated in SH-SY5Y cells, and the mRNA and protein levels of NOX4 were significantly upregulated. After treatment with the miR-92b-3p mimics, the expression of miR-92b-3p was reversed at the NOX4 protein level but did not affect the expression level of NOX4 mRNA, indicating that miR-92b-3p works by inhibiting the translation of NOX4 mRNA rather than by degrading NOX4 mRNA (Figures 6(b)–6(d)). The ROS test results in the cell culture medium showed that the amount of ROS released into the culture medium of SH-SY5Y cells increased after H/R, but after treatment with the miR-92b-3p mimics, this effect was reversed. These results are consistent with alterations in NOX4 protein levels.

The article "miR-92b-3p Exerts Neuroprotective Effects on Ischemia/Reperfusion-Induced Cerebral Injury via Targeting NOX4 in a Rat Model" was retracted in 2023. Reasons: signs of a paper mill; compromised peer review; unreliable results or conclusions.

### 3.7. Exogenous miR-92b-3p Mimics Decreased Apoptosis Induced by H/R in SH-SY5Y Cells

Hoechst staining and flow cytometry was utilized to analyze the effect of H/R exposure on nerve cell apoptosis. Hoechst staining results showed that H/R caused obvious nuclear fragmentation and apoptotic bodies in SH-SY5Y cells, and cotransfection of miR-92b-3p mimics significantly reversed the production of apoptotic bodies. The Hoechst staining apoptosis statistics showed that the apoptosis rate of the control group was approximately 5%. H/R caused an increase in the apoptosis rate to 30%, and intervention with the miR-92b-3p mimics increased the apoptosis rate to 20% (Figures 7(a) and 7(b)). Flow cytometry results showed that the overall (early and late) apoptosis rate of the control group was approximately 15%. After H/R intervention, the overall apoptosis rate was 40%, and intervention with the miR-92b-3p mimics caused an increase in the overall apoptosis rate to 24%, which was essentially consistent with the Hoechst staining results.

### 3.8. Effect of miR-92b-3p Overexpression on Luciferase Reporter Gene Expression

To provide direct evidence of the interaction between miR-92b-3p and NOX4, we constructed the luciferase reporter gene SV40-Luci-NOX4 3′UTR-PolyA (Figure 7(e)). The luciferase activity results showed that H/R significantly upregulated the luciferase activity, and after intervention with the miR-92b-3p mimics, the inhibitory effect of H/R treatment on luciferase activity was significantly reduced, indicating that miR-92b-3p could indeed bind to the untranslated region of the NOX4 gene and inhibit its translation (Figure 7(f)).

The article "miR-92b-3p Exerts Neuroprotective Effects on Ischemia/Reperfusion-Induced Cerebral Injury via Targeting NOX4 in a Rat Model" was retracted in 2023. Reasons: signs of a paper mill; compromised peer review; unreliable results or conclusions.

## 4. Discussion

In this study, we established a model of cerebral I/R injury in SD rats. TTC staining, HE staining, TUNEL staining, and caspase-3 activity detection indicated that the local brain tissue was infarcted, the morphological structure of the brain tissue was destroyed, and cell apoptosis had increased. The mortality rate increased, and the neurobiological function scores ranged from 1 to 4, indicating that the establishment of the cerebral I/R model was successful. To simulate in vivo cerebral I/R injuries, we established a neuronal cell injury model induced by H/R. The results showed that hypoxia for 4 h and reoxygenation for 24 h could successfully induce neuronal cell damage. The activity of caspase-3 and the rate of apoptosis were significantly increased. Moreover, using bioinformatics-related software, we obtained the following results: (1) after cerebral I/R, there were 3 miRNAs (miR-29b, miR-126a, and miR-92b-3p) associated with 11 brain characteristics or brain-rich miRNAs, and their expression levels in brain tissue decreased significantly, while the expression of only one miRNA (miR-92b-3p) decreased in the plasma, which prompted us to focus our attention on miR-92b-3p; (2) NOX4 is a potential target gene of miR-92b-3p; (3) after cerebral I/R, NOX4 expression at the mRNA and protein in brain tissue was significantly increased, which was in the opposite direction of the miR-92b-3p expression, which was in line with expectations; (4) in the H/R injury model, miR-92b-3p expression was significantly downregulated, and NOX4 mRNA and protein expression levels were significantly increased, with ROS levels rising, effects that could be canceled with a miR-92b-3p mimic; and (5) following transfection of nerve cells with a fluorescein reporter plasmid (SV40-Luci-NOX4 3′UTR-PolyA), H/R treatment significantly inhibited luciferase activity, an effect that could be reversed by miR-92b-3p mimics. These results clarified the role and mechanism of miR-92b-3p in cerebral I/R injury for the first time.

Increased generation of reactive oxygen species during cerebral I/R is associated with upregulation of the expression levels of certain oxidase genes and increased activity [30]. In the oxidase system, the active oxygen derived from NOX is the most extensive. The product of NOX is O2.- (NADPH + 2O2 NOX NADPH++H++O2.-). O2.- is extremely unstable, and it quickly turns into H_2_O_2_. The NOX family includes NOX1–5, Duox1, and Duox2 [31, 32]. A large number of studies have shown that NOX-derived active oxygen plays important role in oxidative stress injury in cerebral I/R [33]. Knockout of NOX or the administration of drugs that inhibit NOX activity could significantly reduce the volume of cerebral infarction in mice or rats after I/R and ameliorate nerve function [34]. Recently, the expression levels of the main subtypes of the NOX family (NOX1–4) in brain tissues were screened, and it was found that both NOX2 and NOX4 were upregulated, while NOX1 expression showed no significant changes and NOX3 expression was not detected, suggesting that NOX2 and NOX4 are the main contributors to oxidative stress injury during cerebral I/R in rats [33, 34]. Numerous studies have demonstrated that NOX inhibitors, especially NOX2- or NOX4-specific inhibitors, should be able to ameliorate cerebral I/R-induced oxidative injury [35]. Several NOX inhibitors (such as DPI, apocynin, PR39, Gp91ds-tat, and VAS2870) have indeed been shown to exert protective effects on cerebral I/R injury, but currently, these inhibitors are only used as tools for medicinal applications [8, 18]. Therefore, with NOX4 as the target, searching for drugs against cerebral I/R oxidative injury has broad clinical application prospects.

The article "miR-92b-3p Exerts Neuroprotective Effects on Ischemia/Reperfusion-Induced Cerebral Injury via Targeting NOX4 in a Rat Model" was retracted in 2023. Reasons: signs of a paper mill; compromised peer review; unreliable results or conclusions.

As noncoding short-chain RNAs, miRNAs play an important role in gene expression suppression [36, 37]. Therefore, we preliminarily speculated that the inhibition of NOX4 expression during I/R may be related to the abnormal expression of certain miRNAs. In studies related to cerebral ischemic injury, miRNA chips are currently used to screen miRNAs with abnormal expression in brain tissues [38]. Since there are thousands of reported miRNAs, the amount of information obtained by the miRNA chip is vast, and most studies only focus on the data, while in target gene analysis and prediction stages, there has been little in-depth discussion. To focus on the scope of the research, the present study focused on brain-specific or brain-rich miRNAs because we believe that changes in the expression levels of these miRNAs can more directly reflect cerebral I/R injury. By carefully reviewing published results, 8 brain-specific or brain-rich miRNAs were specified as targeted miRNAs in cerebral I/R injury. Through real-time PCR analysis, we found that 3 miRNAs (miR-29b, miR-126a, and miR-92b-3p) in brain tissue were downregulated, while only miR-92b-3p levels in the plasma decreased noticeably [39]. In the rat model of cerebral I/R injury, only miR-92b-3p was significantly decreased in the brain tissue and plasma. Using the bioinformatics analysis software, we initially speculated that NOX4 is a potential target gene of miR-92b-3p.

In vivo experiments have demonstrated that the direction of miR-92b-3p level change in brain tissue is opposite to the direction of expression change, indicating that miR-92b-3p may inhibit the expression of NOX4. To verify the relationship between miR-92b-3p and NOX4, a neural cell (SH-SY5Y) hypoxic injury model was established to simulate a global I/R injury model. Using this model, we confirmed that miR-92b mimic could block the downregulation of NOX4 expression by H/R and initially determined the inhibitory effect of miR-92b-3p on NOX4 expression.

The article "miR-92b-3p Exerts Neuroprotective Effects on Ischemia/Reperfusion-Induced Cerebral Injury via Targeting NOX4 in a Rat Model" was retracted in 2023. Reasons: signs of a paper mill; compromised peer review; unreliable results or conclusions.

According to the results of bioinformatics analysis, miR-92b-3p mainly functions by binding to a specific sequence of the 3′ untranslated region of NOX4. Therefore, we constructed a luciferin reporter gene in the 3′ untranslated region of NOX4. Using this reporter gene, we found that luciferase activity was significantly reduced after H/R, an effect that could be reversed by overexpression of miR-92b-3p mimic. These results strongly demonstrated that miR-92b-3p could indeed combine with the NOX4 3′ untranslated region to inhibit NOX4 expression. Since miR-92b-3p mimic does not affect the expression level of NOX4 mRNA, miR-92b-3p inhibits NOX4 expression. The effect occurs at the translation level rather than the transcription level.

Collectively, miR-92b-3p may be involved in the occurrence of oxidative stress during cerebral I/R, and its mechanism may be through the inhibition of NOX4 expression, resulting in a significant decrease in NOX4 activity, which eventually leads to oxidative stress injury.

## Figures and Tables

**Figure 1:** Cerebral I/R caused cerebral infarction and neurobiological damage in rats (*n* = 8). (a) Neurological function scores of rats in different groups. (b) Representative pictures of TTC staining of brain tissue sections of rats in different groups (red is a noninfarcted area, and white is an infarcted area). (c) Cerebral infarction volume in different groups. (d) Histopathological changes. Control: control group; sham: sham operation group; I/R: cerebral ischemia/reperfusion group. All the data are presented as the mean ± standard error. ^∗∗∗^*P* < 0.001 vs. the sham group.

**Figure 2:** Changes in the apoptosis of brain tissue cells after cerebral I/R in rats. (a) Representative pictures of TUNEL-positive cells in rat brain tissue, in which dark blue particles are apoptotic cells (×200). (b) Statistical results of TUNEL-positive cells in rat brain tissue (*n* = 5). (c) Caspase-3 activity changes in brain tissues of different groups of rats (*n* = 8). Control: control group; sham: sham operation group; I/R: cerebral ischemia/reperfusion group. All the data are expressed as the mean ± standard error. ^∗^*P* < 0.05; ^∗∗^*P* < 0.01.

The article "miR-92b-3p Exerts Neuroprotective Effects on Ischemia/Reperfusion-Induced Cerebral Injury via Targeting NOX4 in a Rat Model" was retracted in 2023. Reasons: signs of a paper mill; compromised peer review; unreliable results or conclusions.

**Figure 3:** Expression of miRNA-rich brain tissue after cerebral I/R in rats. Control: control group; sham: sham operation group; I/R: cerebral ischemia/reperfusion group; ^∗^*P* < 0.05; ^∗∗^*P* < 0.01.

**Figure 4:** NOX4 functioned as a direct target gene of miR-126a-5p. (a) Analysis of miR-92b-3p targets. (b) Analysis of NOX4 (TECPR2) target miRNA. (c) Sequence analysis of miR-92b-3p and NOX4. (d) The luciferase reporter vector of NOX4-WT or NOX4-MT was cotransfected with NC mimic or miR-92b-3p mimic in 293T cells. After 48 h transfection, the relative luciferase activity was evaluated. SH-SY5Y cells were treated with miR-126a-5p mimic or NC mimic for 48 h. (e) mRNA and (f) protein levels of NOX4 regulated by miR-126a-5p in SH-SY5Y cells measured by qRT-PCR and Western blot. Data are presented as mean ± standard error. ^∗∗^*P* < 0.01. *n* = 6.

**Figure 5:** The expression of miR-92b-3p in brain tissue and plasma and the mRNA and protein levels of NOX4 in brain tissue after cerebral I/R in rats. (a) miR-92b-3p levels in brain tissues of rats. (b) miR-92b-3p levels in the plasma of rats. (c) NOX4 mRNA levels in brain tissues of rats. (d) NOX4 protein expression in rat brain tissues. Control: control group; sham: sham operation group; I/R: cerebral ischemia/reperfusion group; ^∗^*P* < 0.05, ^∗∗^*P* < 0.01, *n* = 6.

**Figure 6:** Exogenous miR-92b-3p mimic decreased NOX4 expression level and oxygen-free radical content. (a) The inhibitory effect of the miR-92b-3p mimic on miR-92b-3p expression. (b) miR-92b-3p expression level. (c) NOX4 mRNA level. (d) NOX4 protein. (e) ROS levels. Control: control group; H/R: hypoxic/reoxygenation group; +mimic: hypoxic/reoxygenation+miR-92b-3p mimic (100 nmol/l) group; +NC mimic: hypoxic/reoxygenation+negative control (100 nmol/l) mimic group; ^∗∗^*P* < 0.01, *n* = 6.

**Figure 7:** Effect of miR-92b-3p mimic on apoptosis and luciferase reporter gene expression induced by H/R. (a) Representative pictures of Hoechst-positive nerve cells (×200). (b) Statistical results of Hoechst-positive nerve cells. (c) Flow cells of nerve cells. (d) Statistical results of flow cytometry of nerve cells. (e) Schematic of the SV40-Luci-NOX4 3′UTR-PolyA plasmid. (f) Statistics of luciferase activity in the different groups. Control: blank control group; H/R: hypoxic/reoxygenation group; + mimic: hypoxic/reoxygenation+miR-92b-3p mimic (100 nmol/l) group; +NC mimic: hypoxic/reoxygenation+negative control (100 nmol/l) mimic group; ^∗^*P* < 0.05; ^∗∗^*P* < 0.01, *n* = 6.

**Table 1:** Primer or gene sequence list.

Gene name Primer or gene sequence
NOX4 Forward:5′-CTTTAGCATCCATATCCGCATT-3′
Reverse:5′-GACTGGTGGCATTGTCACAATA-3′
*β*-actin
Forward:5′-CCCATCTATGAGGGTTACGC-3′
Reverse:5′-TTTAATGTCACGCACGATTTC-3′
U6 Forward:5′-CTCGCTTCGGCAGCACA-3′
Reverse:5′-AACGCTTCACGAATTTGCGT-3′
miR-92b-3p 5′-UCUUUGGUUAUCUAGCUGUAUGA-3′

The article "miR-92b-3p Exerts Neuroprotective Effects on Ischemia/Reperfusion-Induced Cerebral Injury via Targeting NOX4 in a Rat Model" was retracted in 2023. Reasons: signs of a paper mill; compromised peer review; unreliable results or conclusions.

## Data Availability

The data used to support the findings are available from the corresponding author upon request.
